RETRACTED

# Psychological Stress Identification and Evaluation Method Based on Mobile Human-Computer Interaction Equipment

**DOI:** 10.1155/2022/6039789

**Published:** 2022-04-25

**Authors:** Na Zhang

**Affiliations:** Department of Ideological and Political Education, Ulanqab Medical College, Ulanqab, 012000 Inner Mongolia, China

## Abstract

Since the 1980s, the research of artificial neural networks in the field of artificial intelligence has become more and more common. It accepts nonlinear parallel processing, has strong learning and flexibility, and can be used for influencing factor analysis. The ideal power values and triggers are obtained in the Hopfield network model using genetic algorithm, which best avoids the drawbacks of the Hopfield network model instillation learning method. Through the BP of mobile human-computer interaction equipment, hereditary, genetic algorithms, and Hi-PLS regression method in the artificial neural network, the psychological pressure of college students is identified, evaluated, and predicted from three dimensions such as learning, life, and personal events. This makes it possible to understand the current physical and mental conditions of the students in a timely manner, guide to relieve anxiety and fear, and reach a safe psychological level. The three test results are less than 1%, which has high research significance and value.

## 1. Introduction

With the growth of our society and the advancement of our skills in recent years, a great deal of records and data has been accumulated in the course of many example projects on the study of psychological stress. However, these are stored purely for the purposes of database building and are not well used, resulting in a waste of data resources in the psychological research industry. We urgently need an artificial neural network technology to use and analyze human psychological pressure construction data and obtain corresponding laws and conclusions, to provide valuable information for people to study psychological changes. Mobile human-computer interaction equipments are widely used, and products have already entered the market. Mobile human-computer interaction equipments are being further developed to simulate human cognition. Computational intelligence has become an important direction in artificial intelligence through the combination of BP schemes, hereditary methods, and developmental systems. This relatively mature technology is applied to people's physical and mental health to identify and monitor psychological stress.

Recognizing psychological pressure through mobile human-computer interaction equipment, providing reference for review work, and evaluating the dynamics and rationality of psychological pressure can be used to provide guidance for the design of psychological pressure prediction. The introduction of intelligent analysis algorithms can improve the efficiency and level of analysis. At the same time, this study can also provide some basis for the development of mental health education in universities. It is useful for gaining insight into the current conditions and characteristics of people's psychological safety and for promptly identifying and learning about the sources of stress in everyday life. It is helpful to guide them to actively adapt in stressful situations, relieve anxiety and fear, improve their psychological security, and face life and work with a safe and stable state of mind.

RETRACTED

The ability of mobile human-computer interaction equipment to process data offline surpasses traditional human intelligence methods. It uses real-time detection, integration, and knowledge of other disciplines to identify and monitor the movement of psychological pressure.

## 2. Related Work

In the past few years, the evolution of artificial intelligence has permeated all walks of life, and the trend is on a straight upward trajectory. According to Almonacid et al., it is based on the advantages of mobile human-computer interaction equipments in solving complex and nonlinear problems, as well as the high complexity of electrical modeling of CPV equipment. In order to approach different problems related to low-polymer and high-tech polymer photovoltaics, he reviewed mobile human-computer interaction equipments. In addition, he reviews mobile human-computer interaction equipment models to anticipate the main ambient factors influencing properties [1]. Radziszewski presents the results of research in the field of computer knowledge and examines the scope of application of manual network techniques as a tool for construction planning. The computational tests used error back propagation to train the synthetic network, which was based on the geometry of the Roman Collins capital detail. Once the artificial network is successfully trained, it can imitate any other geometric type given [2]. Canziani et al. analyzed their spectral characteristics acquired from these satellite pictures to infer the nutrient status of the shore and generate a real-time tool for investigating the shore lake dynamics, with statistically significant results [3]. Perchiazzi et al. hypothesized that a mobile human-computer interaction equipment could evaluate PEEP tot from traffic and blood pressure tracking during continuous institutional inflation [4]. According to Kiran et al., application of artificial intelligence techniques is combined with a Box-Behnken (BB) design to simulate process parameters for the use of live algae (Arthrospira) spp. for cadmium biosorption [5]. Menino et al. study the relationship between gender affirmation medical intervention and the improvement of the mental health of transgender people. Other potential risk factors associated with transgender specificity should be investigated in future studies [6]. Yuenyongchaiwat suggested that an increased physiological response (i.e., cardiovascular reactivity) to one or more sources of stress may increase the potential risk of developing coronary heart disease (CVD), which includes elevated blood pressure (BP) or high blood pressure. The aim of the research was to check to see whether the central coronary response to psychological stressors remained a significant predictor of CVD in Asian Thai participants with initially normal BP at 40-month follow-up. After these participants rested, their blood flow parameters, mental arithmetic, language tasks, and parameters related to cold stress tasks were measured [7]. Wang et al. developed a model for wind farm power range forecasting using multiple output characteristics based on BP nets and proposed an optimal guideline that takes into account information about the forecasting interval. The model was then analyzed using an improved particle swarm optimal (PSO) algorithm for modelling [8]. These studies have great reference value for this article, but the time span of related studies is small, and the sample size is insufficient, which leads to certain problems in the results.

RETRACTED

## 3. Psychological Pressure Recognition Method of Mobile Human-Computer Interaction Equipment

The mobile human-computer interaction equipment model originated from the human central nervous system [9]. It simulates the operation of the central nervous system of the human brain, using a series of input data to adaptively calculate or predict output data. This computational step is akin to the human learning curve, resulting in an adaptive process. It adopts nonlinear concurrent treatment and is highly adaptive and adaptive, allowing it to be used for impact element profiling. The following will introduce the typical neural network model of each development period.

1. M-P model

In the 1840s, some psychologists first proposed the MP model to simulate the human neural network, such as the application of data collection, after in-depth study of the neural network of the human brain, as shown in Figure 1. The MP model introduces the concept of neurons for the first time and regards neurons as a binary key, and different combinations of neurons can be used to process various logical operations. It consists of three parts, namely, weighted calculation, linear dynamic system, and nonlinear function mapping [10].

(2) Hopfield network model

In the 1980s, a California Institute of Technology professor proposed a single-mode network model and called it the Hopfield network model [11]. It is mainly used in voltage testing and has a significant guarantee for voltage safety performance. As shown in Figure 2, the Hopfield model introduces the network energy function for the first time and brings the neuron entry and exit latency into a new network, using the needle learning process to determine the “metric and threshold” of the network item. The neural network is designed in one way, but this method keeps the parameters and boundaries of the network unchanged. The collaborative memory function of the Hopfield network model accurately describes human behavior. An important feature of Hopfield network is that it can play the role of joint memory, that is, as joint memory. When the network load is determined by learning and training, even if the input data is incomplete or the components are incorrect, the network can provide complete output results through collaborative memory. After the professor proposed this model, many people tried to expand it, hoping to design a network model closer to the characteristics of the human brain.

(3) Boltzmann machine network model

In the second half of the 1880s, computer scientists proposed a Boltzmann machine network model on the basis of the artificial neural nerve model. As illustrated in Figure 3, the Boltzmann machine lattice model is mainly superior to the fixed determination of Hopfield lattice model in weight distribution [12]. The computer scientist simulated annealing algorithm randomized the weight distribution to the artificial nerve model. It is a typical random artificial nerve model. The Boltzmann machine network model finds the answer through the simulated annealing process, which makes the training time of the neural network longer.

(4) RBF nerve model

In the second half of the 1880s, computer scientists proposed the Boltzmann machine network model on the basis of the artificial nerve model [13], and theoretically, the indivisible problem can be derived. As RBF network theory can be derived for the input layer input signaling composition of the function, the joint wastes between both the input and implicit tiers are an inseparable issue. The hidden layer performs the image of the image cast of the input resources, and the outgoing list is the most important one. The optimization parameters that RBF needs to learn include the center of gravity base of the function output layer and the adjustment of the excitation function. The parameters slow down the learning rate through a linear optimization strategy. Different types include direct selection path, random center path, control center path, and small square path. Taking the integration method as an example, learning it involves two steps. The first step is a noncustodial learning process, by defining the basic functions of a layer and a large area; the second phase is a controlled learning process, which can analyze the degree of integration from hiding to output [14]. A very important reason is that its hidden part is close to the network, without learning and avoiding the continuous interlayer transmission process in the hierarchical network. RBF neural systems are an integral part of the results of the exercise and have been successfully used for sequencing, dehydration function approximation, model implementation of model based information handling systems, data analysis of temporal variables, error diagnosis, and fault design, as illustrated in Figure 4.

(5) New combined neural network model

Since the 21st century, in a bid to get over the drawbacks of local excellence arising from the long training time of a single steering system, experts and scholars have begun to use the method of combining neural networks. Experts and scholars have begun to use the method of combining neural networks to reason, intervene and diagnose the system, and have achieved good results in answering different questions for the same knowledge structure. British data scientists have absorbed the advantages of this series of biological evolutionary algorithms and combined the genetic algorithm with the Hopfield network model. He used hereditary techniques to obtain the ideal pair of weapons and triggers in the Hopfield web system model, which best avoids the drawbacks of the Hopfield web system model's indoctrination learning method. Some experts use the membership theory in fuzzy mathematics combined with BP neural network to establish a new type of fuzzy web system model combination model, which can not deal with the shortcomings of fuzzy problems [15].

RETRACTED

Artificial neural networks have lots of features that capture explicitly or otherwise the advantages or operating principles of them such as bionic properties, properties of massively combined parallel computing, nonlinear properties and teacher learning, extensive features, self-adaptive features, worldwide features, and error tolerant and unifying features. The most important of these is the Hi-PLS, whose method is mainly suitable for regression modeling of multiple groups of independent variables and a group of dependent variables. In the process of actual data analysis, PLS regression is very effective in the modeling process of multivariate psychological stress test.

### 3.1. BP Neuro Nets

BP neuro net is a characteristic response to artificial nerves. The key elements of this system are the automatic traffic of data and the propagation of bugs in the background. In the bypass, the input signal is controlled layer by layer, and the input switch is hidden from input to output. The condition of individual cells in each layer impacts only the condition of cell elements in the next layer [16]. It is shown in Figure 5.

BP nets are many layer networks. In addition to the import and export tiers, there are also embedded pairs of tiers. BP neural network adopts the method of error back-propagation to reduce errors, but it has limitations, requires many parameters, and is easy to fall into local optimum. The amount of concealed tiers is variable and can be an integer greater than or equal to 1. It is worth noting that the network uses the BP algorithm to adjust the weights. As shown in Figure 6, it is a BP neural model with *n* private levels. As can be seen from the figure, in the BP neural model, data information is spread layer by layer, from the input layer to the hidden layer. In the corresponding weight network training process, along the direction of error reduction, the output layer gradually passes through the hidden layer. The neural web powers are corrected in advance, and through repeated learning and training, the error eventually becomes smaller and smaller to reach the study scenario [17].

Generally speaking, the BP structure has the following characteristics: First, the BP structure is composed of multiple layers, the neurons in the same layer are independent of each other, and the layers are connected. It is the multilayer design of neural networks that allows BP nets to mine more data from the entry tiers and to undertake more complex modeling tasks. Second, the pass along of the BP nets has to be continuously trivial; third, the BP algorithm is used for learning [18].

Its unique BP structure design includes the number of tiers of the web, the count of entry level points, the capacity of the return nodes, the capacity of the back output nodes, the capacity of the hidden nodes, and the transfer function, learning, training function, and parameter definition. This area is introduced in the following BP test, combined with pressure, that is, a detailed description of the pressure response analysis.  Figure 7 shows the human stress response system.

Tables 1 and 2 are the numbers, thresholds, and output performance that need to be stored in the fields and attributes of the neuron class.

The error is judged by the artificial neuron class array and neuron class field, and the error is kept within 1%, which can be better analyzed and judged.

RETRACTED

### 3.2. Genetic Algorithm

Genetic algorithm is to integrate problem solving into molecules. Genetic algorithm overcomes the shortcoming of being stuck in an infinite loop and is a global optimization algorithm. At the same time, the molecular algorithm is an exact solution, not a true solution. An exact solution is infinitely close to the true solution but never reaches the true solution. It takes the TSP problem as an example to show that there is no simple and direct solution. If it want to solve it correctly, use the return method, which increases the complexity a lot [19].

### 3.3. Hi-PLS Regression Method

PLS regression uses the principle of main part analysis to compress several *X* and *Y* into multiple parts (*X* which answers to main element *U* and *Y* which answers to main element *V*); then by means of typical relating principle, the association between *X* and *U* can be obtained, and the relationship between *Y* and *V* can be analyzed, and combined with the angle of linear progression principle, the analysis of the interaction between *X* and *V* is used to study the association between *X* and *Y*.

Since the PLS regression method was proposed, the method has been greatly developed in theory and practical application [20]. One of the most important theories and research results is the proposal of the Hierarchical Partial Least Square (Hi-PLS) model [21]. This method is mainly suitable for the regression modeling of multiple independent variables and a set of dependent variables in the actual data analysis process. PLS regression is very effective in the process of multivariate modeling. It represents a straight line in the mathematical model. This results in a low linear regression prediction rate for the monomial, but if there are too many independent variables, the model results obtained will be very complicated and difficult to interpret and analyze. Therefore, there is an urgent need to find a new, reasonable, and effective method that can reduce the huge number of independent variables to a number that is easy to handle. The Hi-PLS regression method, for example, can reduce a huge number of independent variables to a manageable number. However, if it simply delete some independent variables, the way to select some independent variables for modeling is obviously unreliable. This may cause the loss of important information, leading to the construction of wrong models and false interpretations and analyses [22].

## 4. Psychological Stress Recognition Experiment Based on Artificial Reactive Honeypot Theory

### 4.1. BP Nets

In the process of BP net modeling, BP involves the setting and adjustment of a large number of related parameters. In addition, there are other specific parameter settings such as implicit layer, delivery function of the export layer, and learning function. It is difficult to judge directly which combination method is more appropriate. The research adopts the “trial and error method,” which judges by comparing the mean square error of each model through different combinations of various parameters. The BP neural network adopts a supervised learning method. Therefore, when we apply the model to solve practical problems, a training data set is one of the necessary prerequisites. Designing a BP neural network model mainly includes the amount of web tiers, the quantity of injection tier knots, the quantity of output tier knots, and the quantity of implicit tier knots, as well as the transfer function, learning function, training function, and training parameter settings [23].

RETRACTED

The number of the entry level nodes depends on the size of the input vector. The output vector is actually the expected output provided for the BP neural network. A BP neural network can have multiple outputs, and the output can be either a numerical variable or a linguistic variable. If there are *m* categories, *m* neurons can be used as the output. The research intends to use the medical consortium performance score as the output value, and the number of nodes in the output layer is 1.

The choice of the nodes of the latent levels has a strong influence on the training performance of the BP neural net model. Generally speaking, a large number of hidden layer nodes can optimize the performance of the model, but it may also lead to too long training time. There is still no good idea to determine the actual amount of nodes in the latent floor, and a common method is called the “ patchwork method.” The general approach is to use empirical formulas to give estimates, and these estimates can usually be used as the initial values of the trial and error method. Based on this, it can adjust itself during the model training process [24].

The transfer function, also known as the “activation function,” is a key component of the BP model, and the transfer function must be continuous and differentiable.

The learning of the BP model belongs to supervised learning, and the data set that needs to have an output value is called the learning sample set. Modifying the weights down the opposite order of the error performance function belongs to the most rapid descent method [25].

The training function needs to be learned and trained separately to select the best combination form.

RETRACTED

The BP neural network model uses an iterative update method to determine the weight, so the network needs to determine an initial value. The initial value is usually defined as a small nonzero random number. The empirical values are positive and negative, to which *m* is the count of injection layer knots. But this method also has a certain degree of subjectivity and uncertainty. Generally, in the process of modeling, the initial weights are not defined deliberately but are given arbitrarily by the software. However, if this method is adopted, it is easy to cause the unreproducibility of the network, which is also one of the shortcomings of the BP net. Based on the above factors, this study sets the number of network loop training to 50 times, trains each candidate model 50 times, and selects the one with the smallest root mean square error for final screening.

Before performing neural tree forecast, the tree must be trained, and the database has the ability of recall and evaluation through the process of training.

1. *Web Priming*. Based on the entry-output order of the proposed system (*X*, *Y*), determine the node count of the *m*th entry list of the neural model, the hid list of nodes is l, and the output list of nodes is *n*. Initialize the joint weights between the neurons of the entry and output layers are *w*_*ij*_ and *w*_*jk*_. It initializes the hidden layer threshold to *a* and the output layer threshold to *b* and specifies the learning rate and activation function of the neuron
2. *Hidden Layer Export Function Is Applied*. The output of the hidden layer *H* is calculated based on the input variable *X*, the *w*_*ij*_ joint power between the input and hidden layer, and the boundary *a* of the concealed layer. The formula is as follows:

(1) $$\begin{array}{c} H_{j}=f\left(\overset{m}{\underset{1}{\sum }}w_{ij}-a\right)j=1,2\cdots ,l, \end{array}$$

where *f* is the implied floor excitation feature, which has various expressions, and the ones used in this paper are:

(2) $$\begin{array}{c} f\left(x\right)=\frac{1}{1+e^{-x}}. \end{array}$$

1. *Input Method Calculation*. The predicted output *O* of the BP neural network is calculated based on the hidden level input *H* with the connection weights and the gate value *b*, which is given by:

(3) $$\begin{array}{c} O_{k}=\overset{l}{\underset{1}{\sum }}H_{jwjk}-b_{k}k=1,2,3,\cdots ,n. \end{array}$$

(2) *Error Calculation*. According to the predicted output *O* and expected output *Y* of the neural network, calculate the prediction error *e* of the BP neural network:

(4) $$\begin{array}{c} e_{k}=Y_{K}-O_{K}. \end{array}$$

(3) *Weight Update*. Update the *w*_*ij*_ and *w*_*jk*_ networks according to the error *e*, where *η* is the learning rate. The formula is as follows:

(5) $$\begin{array}{c} W_{ij}=W_{ij}+\eta H_{j}\left(1-H_{j}\right)x\left(i\right)\overset{m}{\underset{k=1}{\sum }}w_{jk}e_{k}i=1,2,\cdots ,m;j=1,2,\cdots l, \end{array}$$

(6) $$\begin{array}{c} W_{ij}=W_{ij}+\eta H_{j}e_{k}j=1,2,\cdots ,l;k=1,2,\cdots ,n. \end{array}$$

(4) *Threshold Update*. Update node thresholds *a* and *b* according to error *e*

(7) $$\begin{array}{c} a_{j}=a_{j}+\eta H_{j}\left(1-H_{j}\right)x\left(i\right)\overset{m}{\underset{k=1}{\sum }}w_{jk}e_{k}j=1,2,\cdots ,l, \end{array}$$

(8) $$\begin{array}{c} b_{k}=b_{k}+e_{k}k=1,2,\cdots ,n. \end{array}$$

(5) Judge whether it is over, if not, go back to Step 2.

RETRACTED

### 4.2. The Main Function of Genetic Algorithm

The genetic algorithm process is range value.

For the first step, it randomly initializes the population.

For the second step, it calculates the fitness value of the population and finds the most individual from it.

For the third step, it will choose the operation.

For the fourth step, it will cross-operate.

For the fifth step, it will mutate operation.

For the sixth step, it judges whether the evolution is over, if not, it returns to the second step.

When selecting according to the function design, the fitness value is proportional to the probability of inheritance to the next generation. In order to maximize the fitness value, the reciprocal value of the total path length is used as the fitness value. According to the unique method of genetic algorithm, the weight is optimized, and the optimized network weight is used as the current layer to continue back propagation, and this step is repeated until the end of the training [26]. At home and abroad, there are physical subhealth caused by excessive stress, such as karoshi, depression, and other symptoms; severe cases are fatal, and mild cases affect work and life. This paper mainly analyzes the large group of college students in China which is targeted. The genetic algorithm is used to test the differences in psychological stress and psychological elasticity of Chinese college students. The comparison of the test results is shown in Figure 8.

Figure 8 shows that the independent sample *t*-test of psychological stress factors of college students of different genders found that there is no significant difference between men and women in the total stress scores of college students. It conducts independent tests on the psychological flexibility and various factors of college students of different genders. From the analysis of various dimensions of mental toughness, male and female college students have significant differences in resilience, boys are higher than girls, and there are significant differences in intensity and optimism. This shows that male college students tend to be more calm than female college students when facing challenges. The differences in psychological stress and psychological flexibility of college students of different genders are directly proportional.

RETRACTED

From the perspective of the overall pressure of college students, the only child has a significant impact on the pressure of college students. In the three dimensions of learning, social, and family pressure, nononly children scored significantly higher than nononly children in terms of personal stress, academic stress, and negative life events. Specifically, non-only-child college students are more stressed than only-child college students. As shown in Figure 9, whether the student is an only child is tested. The results show that in terms of total flexibility, there are obvious psychological differences among only children. The large psychological pressure of the nononly child is directly proportional to the test of the difference in psychological flexibility. For example, its study pressure, life pressure, family pressure, and social pressure will be greater than the only child pressure.

With the development of society, whether it is people's life pressure or work pressure has been clearly displayed, mainly due to living costs, education costs, work intensity, etc., such as karoshi, depression, and other symptoms. In order to better determine the weight of the three dimensions of psychological resilience in the total mediating effect, it is necessary to continue to analyze the mediating effects of resistance, strength, and optimism. The return of optimism, to analyze whether the stress of college students is affected by their tenacity, strength and optimistic return psychology. As shown in Figure 10, the mediating effects of tenacity, strength, and optimism were 23.2%, 24.3%, and 15.9%, respectively. It can be seen that the mediating effect of college students' psychological resilience on college students' pressure and psychological security. Among them, tenacity accounts for the highest proportion, followed by strength, and optimism is the weakest.

### 4.3. Hi-PLS Regression Method

In 1996, based on this simple and feasible multivariate hierarchical modeling idea, some researchers proposed Hi-PLS regression, which is famous for its suitability for massive data modeling. After importing the data into the software, it is configured as required. By default, the software selects the nonhierarchical PLS model for analysis and automatically selects the optimal number of components according to indicators such as cross-validity [27]. The steps of applying Hi-PLS regression modeling can be simplified as shown in Figure 11.

RETRACTED

Before modeling, the data needs to be standardized. For convenience, we still denote the standardized data matrix as *E* and *F*. Assuming that according to certain criteria, the independent variable *E* can be divided into *p* blocks, namely:

(9) $$\begin{array}{c} E=\left(E_{1},E_{2},E_{3},\cdots \cdots ,E_{P}\right). \end{array}$$

Each block *E*_*i*_(*i* = 1,2,3,4,5, ⋯, *p*) contains *pi* independent variables, namely:

(10) $$\begin{array}{c} E_{i}=\left(E_{i1},E_{i2},E_{i3},\cdots \cdots ,E_{iP}\right). \end{array}$$

After the preparatory work is done, Hi-PLS regression modeling is carried out next. The first step is to establish a base model, divide multiple independent variable sets into several blocks *E*_*i*_(*i* = 1, 2, 3, ⋯, *p*), and establish a PLS regression model of each independent variable block and dependent variable *F* in turn. According to the principle of cross validity, the corresponding principal component *t*_*i*1_, *t*_*i*2_, *t*_*i*3_, *t*_*i*4_, ⋯*t*_*im*_, (*i* = 1, 2, 3, ⋯, *p*) is extracted. Here, *m*_*i*_ is the number of principal components in *E*_*i*_ extracted. The second step is to establish a top model (top model), that is, perform PLS regression on the principal components *t*_*i*1_, *t*_*i*2_, *t*_*i*3_, *t*_*i*4_, ⋯*t*_*im*_, (*i* = 1, 2, 3, ⋯, *p*) of each block *E*_*i*_(*i* = 1, 2, 3, ⋯, *p*) extracted again with the dependent variable. Similarly, according to the principle of cross-validity, the corresponding principal components are extracted. In the third step, the linear combination of each block *E*_*i*_(*i* = 1, 2, 3, ⋯, *p*), that is, the principal component *t*_*i*1_, *t*_*i*2_, *t*_*i*3_, *t*_*i*4_, ⋯*t*_*im*_, (*i* = 1, 2, 3, ⋯, *p*) obtained from the bottom model, is brought into the top model, and the linear regression formula of the dependent variable *F* related to *E*_*i*_(*i* = 1, 2, 3, ⋯, *p*) can be obtained.

In the process of PLS modeling, the predictive ability of the model is usually judged based on the cumulative cross-validity of the extracted components [28]. If the following factors cannot provide further logical information to explain the difference, many amendments will destroy the understanding of basic statistical properties, leading to the end of false assumptions.

In the process of PLS regression modeling, all sample points are divided into two parts. The first part is to remove the collection of all sample points (containing *N* − 1 sample points) of a certain sample point *j*, use *N* − 1 sample points, and use a principal components to fit a PLS regression formula. In the second part, the excluded ones are brought into the previously fitted PLS regression formula, and the fitted value of *f*_*j*_(*j* = 1, 2, 3, ⋯, *d*) on the sample point *i* is obtained *f*_*aj*(−*i*)_. For each *i* = 1, 2, ⋯, *n*, repeat the above steps, then the sum of squared prediction errors of *f*_*i*_ can be defined as *S*_press,*aj*_; there is

(11) $$\begin{array}{c} S_{\text{press},aj}=\overset{n}{\underset{i=1}{\sum }}{\left(f_{ij}-f_{aj\left(-i\right)}\right)}^{2}. \end{array}$$

Defining the sum of squared prediction errors of *F* as

(12) $$\begin{array}{c} S_{\text{press},a}=\overset{a}{\underset{j=1}{\sum }}S_{\text{press},aj}. \end{array}$$

If the stability of the PLS regression formula is poor and the error is large, it will be more sensitive to changes in sample points. The influence of this disturbance error will increase the value of *S*_press,*a*_.

RETRACTED

At this time, the predicted value is *f*_*aji*_, and the sum of squared errors of *f*_*i*_ is *S*_*ss*,*aj*_, and there is

(13) $$\begin{array}{c} S_{ss,a,j}=\overset{n}{\underset{i=1}{\sum }}{\left(f_{ij}-f_{aji}\right)}^{2}. \end{array}$$

The sum of squared errors of the definition is *S*_*ss*,*a*_, and there is

(14) $$\begin{array}{c} S_{ss,a}=\overset{d}{\underset{j=1}{\sum }}S_{ss,aj}. \end{array}$$

Among them *S*_press,*a*_ > *S*_*ss*,*a*_, *S*_*ss*,*a*_ < *S*_*ss*,*a*−1_, which then compares *S*_*ss*,*a*−1_ and *S*_*ss*,*a*_. Therefore, in the modeling process, it is hoped that the ratio of *S*_press,*a*_/*S*_*ss*,*a*−1_ can be as small as possible. In the SIMCA-P software, specify *S*_press,*a*_/*S*_*ss*,*a*−1_ ≤ 0.95^2^, that is, when

(15) $$\begin{array}{c} \int S_{\text{press},a}\leq 0.95\int S_{ss,a-1}. \end{array}$$

It is believed that adding component *t*_*a*_ is effective, and vice versa, it is ineffective. In addition, there is an equivalent definition: cross-validity. For each dependent variable *f*_*k*_, it can define:

(16) $$\begin{array}{c} Q_{a}^{2}=1{-}_{S_{ss,\left(a-1\right)k}}^{S_{\text{press},ak}}, \end{array}$$

For all dependent variable *F*, the cross-validity of component *t*_*a*_ can be defined as

(17) $$\begin{array}{c} Q_{a}^{2}=1{‐}_{\overset{d}{\underset{k=1}{\sum }}S_{ss,\left(a-1\right)k}}^{\overset{d}{\underset{k=1}{\sum }}S_{\text{press},ak}}=1{-}_{S_{ss,a-1}}^{S_{\text{press},ak}}. \end{array}$$

Applying cross-validity to measure the marginal contribution of *t*_*a*_ to the accuracy of the prediction model, there are two criteria.

(18) $$\begin{array}{c} Q_{a}^{2}\geq \left(1-0.95^{2}\right)=0.0975, \end{array}$$

(19) $$\begin{array}{c} \frac{S_{\text{press},a}}{S_{ss,a-1}}\leq 0.95^{2}. \end{array}$$

For *k* = 1, 2, 3, ⋯, *m*, at least one *k* is *Q*_*a*_^2^ ≥ 0.0975. At this time, adding component *t*_*a*_ will significantly improve the prediction accuracy of at least one dependent variable *f*_*k*_. Therefore, it can be considered that adding component *t*_*n*_ is obviously effective. In summary, the judgment of the PLS regression model needs to be considered in conjunction with *R*^2^ insertion and *Q*^2^. At present, there is no fixed unified standard. Generally speaking, it can refer to two conditions: one is *R*^2^ > *Q*^2^, where *Q*^2^ > 0.5 is enough and *Q*^2^ ≥ 0.9 indicates that the model built is excellent; the second is that the difference between *R*^2^ and *Q*^2^ should not be too large (preferably *R*^2^ − *Q*^2^ < 0.3).

RETRACTED

## 5. Discussion

To recognize and evaluate a person's psychological distress through mobile human-computer interaction equipment, it is generally necessary to express personality characteristics and mood swings related to heart rate, blood pressure, exercise volume, etc. It is also possible to compare different behaviors to judge a person from their thinking. It first determines the reason for the change in behavior and provides information to make a decision. Secondly, it can assess the differences and benefits and advantages of learning experience or personality characteristics and assess the level of development of the child. The third is to provide solid and complete human resources. Fourth, it recognizes the differences between individuals and then predicts the individual differences that may exist in the next individual project or predicts the possibility of success in a specific field in the future. Fifth, individuals can evaluate anxiety, improve their mental health, and understand how to prevent and treat mental illness. It also guides people how to adjust their quality of life and improve their quality of life to understand their mental health.

Because the number of blocks is far less than the total number of original independent variables, and blocks have their specific meaning, compared with traditional PLS regression, Hi-PLS regression has a stronger ability to comprehensively summarize information. Its advantages are more obvious in the process of high-dimensional data analysis and modeling.

## 6. Conclusions

The article studies whether three factors, environment, individual, and economy, can lead to the formation of realistic pressure. Environmental factors include social, economic, and family uncertainties; organizational factors include life cycles such as social structure, social roles, and leadership personality; personal factors include family conditions, personality characteristics, and mental states. Appropriate pressure is conducive to the enthusiasm of work, but long-term stress is not conducive to the healthy development of the body, and it is easy to be in a subhealthy state, such as depression, human immune decline, and other symptoms, which affect work. For example, with symptoms such as a decline in human immunity, people are prone to death from overwork and depression, mild cases affect work, and severe cases threaten life safety.

RETRACTED

## Figures and Tables

**Figure 1:** Topological structure diagram of the M-P model.

**Figure 2:** Topological structure diagram of the Hopfield network model.

**Figure 3:** Topological structure diagram of the Boltzmann machine network model.

**Figure 4:** RBF net model topology structure diagram.

**Figure 5:** BP algorithm flow chart.

**Figure 6:** BP network structures.

**Figure 7:** System model diagram of human body pressure response.

**Figure 8:** The test results of the difference in psychological stress and psychological bombardment among college students of different genders.

**Figure 9:** The test result of the difference in psychological pressure and psychological flexibility for nononly children.

**Figure 10:** Path diagram of the mediating effect of college students' stress, psychological resilience, and psychological security.

**Figure 11:** Schematic diagram of Hi-PLS regression modeling.

**Table 1:** Artificial neuron class field and attribute description table.

Content	Field name	Attribute name	Type	Restrictions
Numbering	artificialNer ronldentifier	ArtificialNer ronldentifier	String	The number starts with “HAN” and “OAN.” The length range is 4 to 10 digits. The text “-1” means that the data is empty or wrong
Range value	thresholdVal	ThresholdValtue	Float	A decimal greater than or equal to -1 and less than or equal to 1
Output	Output	Output	Float	None

**Table 2:** Description table of artificial neuron class array.

Content	Weight array	Input value array
Array name	NeuronWeight	NeuronInput
Array type	Double	Uint
Array size	Scalable in size	Scalable in size
Restrictions	Integer arrays bigger than or similar to 0	Integer arrays bigger than or similar to 0

## Data Availability

Data sharing is not applicable to this article as no datasets were generated or analyzed during the current study.
